The article "MiR-519d targets HER3 and can be used as a potential serum biomarker for non-small cell lung cancer" was retracted in 2025. Reasons: errors in the images; plagiarized images; overlap with other authors' work.

# MiR-519d targets HER3 and can be used as a potential serum biomarker for non-small cell lung cancer

**DOI:** 10.18632/aging.102908

**Published:** 2020-03-13

**Authors:** Aili Wang, Hongxia Zhang, Jinxiang Wang, Shuming Zhang, Zhenyang Xu

**Affiliations:** 1 Department of Respiratory and Critical Care Medicine, Beijing Luhe Hospital, Capital Medical University, Beijing 101100, P.R. China

**Keywords:** serum biomarker, miR-519d, non-small cell lung cancer, HER3

## Abstract

Development of specific serum biomarkers is essential to improve diagnosis and prognosis of non-small cell lung cancer (NSCLC). Here, we show that serum and tissue levels of miR-519d are significantly decreased in NSCLC patients. The low expression of miR-519d is associated with lymph node metastases, clinical stage, and a poor prognosis in NSCLC patients. In addition, ROC analysis demonstrated that the serum miR-519d levels can distinguish NSCLC patients from healthy controls. MiR-519d inhibits proliferation, migration, and invasion by lung cancer cells, indicating that it may function as a tumor suppressor in lung cancer. Furthermore, our data demonstrate that HER3 is a target gene of miR-519d in lung cancer cells, and show that by targeting HER3, miR-519d inhibits the PI3K/Akt pathway. These findings demonstrate that the miR-519d levels are decreased in serum and tumor tissues of NSCLC patients, and indicate that miR-519d regulates NSCLC progression by targeting HER3. MiR-519d could potentially serve as a novel serum biomarker for NSCLC.

## INTRODUCTION

Lung cancer is one of the most common malignant tumors, and a leading cause of cancer related death [1, 2]. Approximately 85% of all lung cancer patients have non-small cell lung cancer (NSCLC) [3]. Most NSCLC tumors are advanced at the time of initial diagnosis, cannot be treated by radical surgery, and are treated only with palliative treatments [4].

Peripheral blood samples from NSCLC patients are the most readily available clinical specimens and can be obtained in a minimally invasive manner [5]. Only small histological or cytological samples can be usually obtained from patients with advanced NSCLC, since these patients are unable to undergo a surgical treatment; however, these samples are usually insufficient for detection of molecular markers [6, 7]. Therefore, development of specific assays for biomarker detection in peripheral blood samples would be of a great significance for NSCLC patients.

Human epidermal growth factor receptor 3 (HER3/ErbB3) is a member of the human epidermal growth factor receptor family [8]. HER3 activates and regulates downstream signaling pathways through the ligand-dependent and ligand-independent dimerization [9]. HER3 has become a potential candidate for tumor therapy in NSCLC and breast cancer patients [10]. However, due to the lack of effective biomarkers, the use of HER3 for NSCLC therapy has been limited [11].

MicroRNAs (miRNAs) are small noncoding RNAs that play a negative role in regulating gene expression [6, 12]. MicroRNA expression is often increased in human malignant tumors, resulting in increased tumor growth, invasion, and metastasis [12, 13]. An abnormal expression of miR-519d has been found in various tumors, including gastric, prostate, and colorectal cancer [14–16]. In prostate cancer, reduced levels of miR-519d have been associated with increased prostate cancer cell proliferation [15]. In addition, previous studies have indicated that the miR-519d expression is decreased in lung adenocarcinoma [17] and NSCLC tissues [18]. However, the underlying mechanisms are incompletely understood, and the miR-519d function in NSCLC is not known.

In this study, we analyzed the expression of miR-519d in NSCLC tissues, and investigated its role in NSCLC progression.

## RESULTS

### MiR-519d levels are decreased in serum and tumor tissues of NSCLC patients

First, we evaluated the miR-519d levels in serum and tumor tissues of NSCLC patients. Compared with healthy controls (1±0.68), the serum miR-519d levels were significantly decreased in NSCLC patients (0.34±0.15) (Figure 1A). In addition, the serum levels of miR-519d were significantly decreased in NSCLC patients of clinical stages II-III-IV (Figure 1B). As shown in Figure 1C, the miR-519d expression was also reduced in tumor lung tissues of NSCLC patients (0.36±0.22) compared to adjacent noncancerous tissues (1±0.62). These data suggest that miR-519d might function as a tumor suppressor gene in NSCLC, and its decreased expression promotes NSCLC development.

**Figure 1:** **MiR-519d expression is decreased in serum and tumor tissues of NSCLC patients.** (**A**) Serum miR-519d levels in NSCLC patients. (**B**) Serum levels of miR-519d in NSCLC patients of clinical stages II-III-IV. (**C**) The expression of miR-519d in tumor lung tissues of NSCLC patients compared to adjacent noncancerous tissues. ^***^p<0.001 vs. control.

### Correlation of serum miR-519d levels with NSCLC clinicopathological characteristics

We evaluated the clinical correlation between serum miR-519d levels and the clinicopathological characteristics of NSCLC patients. Based on the mean expression of serum miR-519d, 130 NSCLC patients were divided into a high expression group (>16.06-fold) and a low expression group (≤16.06). As shown in Table 1, the serum miR-519d levels correlated with the histological grade (p = 0.012), lymph node metastases (p = 0.005), distant metastases (p = 0.035), and clinical stage (p = 0.004). However, no significant correlation was identified between the serum miR-519d levels and patients’ sex, age, tumor size, and histology type (all, p > 0.05).

**Table 1:** Correlation between miR-519d serum levels and clinicopathological variables of NSCLC patients.

**Variable**	**Number**	**Low**	**High**	**P value**
**Age**				0.786
**<60**	55	27	28	
**≥60**	75	39	36	
**Sex**				0.573
**Male**	85	46	39	
**Female**	45	24	21	
**Tumor size**				0.324
**<5 cm**	92	46	46	
**≥5 cm**	38	20	18	
**Histological grade**				0.012
**I**	80	45	35	
**II-III**	50	32	18	
**Histological type**				0.574
**Adenocarcinoma**	40	17	23	
**Squamous**	90	46	44	
**Lymph node metastasis**				0.005
**Yes**	35	17	18	
**No**	95	46	49	
**Distant metastasis**				0.035
**Yes**	34	15	19	
**No**	96	38	48	
**Clinical stage**				0.004
**I-II**	86	46	40	
**III-IV**	44	17	27	

### Serum miR-519d levels can distinguish NSCLC patients from healthy controls

Next, we investigated whether the serum miR-519d level might serve as a potential biomarker to screen NSCLC patients from healthy controls. ROC analysis demonstrated that the serum miR-519d expression could distinguish NSCLC patients from healthy controls, with an AUC of 0.855 (95% CI: 0.803-0.908; P<0.0001). When the cut-off value was 0.22, the sensitivity and specificity were 98.1% and 91.8% (Figure 2).

**Figure 2:** **ROC analysis demonstrating that serum miR-519d levels can distinguish NSCLC patients from healthy controls.**

### Serum miR-519d level is an independent prognostic factor for NSCLC patients

Importantly, significantly shorter overall survival rates were found for NSCLC patients with low miR-519d serum levels compared to patients with high serum. miR-519d levels (*p* = 0.004, Figure 3). Furthermore, univariate and multivariate analyses were carried out to evaluate whether the serum miR-519d expression could be used as an independent biomarker. As shown in Table 2, serum miR-519d expression was an independent prognostic biomarker for the overall survival of NSCLC patients.

**Figure 3:** **Kaplan-Meier curves stratified according to serum miR-519d levels.**

**Table 2:** Univariate and multivariate analyses of serum miR-519d as an independent prognostic biomarker.

**Variable**	**Univariate analysis**		**Multivariate analysis**	
	**HR**	**P value**	**HR**	**P value**
**Age**	1.423	0.342	-	-
**Sex**	1.213	0.578	-	-
**Tumor size**	1.785	0.123	-	-
**Histology type**	1.254	0.187	-	-
**Histological grade**	3.243	0.021	3.132	0.024
**Lymph node metastasis**	4.231	0.004	3.876	0.007
**Distant metastasis**	2.765	0.032	2.432	0.043
**Clinical stage**	3.765	0.008	3.425	0.012
**Serum miR-519d expression**	3.845	0.004	3.635	0.002

### HER3 is a target gene of miR-519d

To identify the target gene of miR-519d, we used the TargetScan, and found a conserved binding site for miR-519d in the 3’ UTR of HER3 (Figure 4A). Dual luciferase reporter assay showed that the relative luciferase activity of pmirGLO-HER3-3’UTR was significantly suppressed by miR-519d, but no changes were found with the mutated HER3-3’UTR (Figure 4B). Transfection of miR-519d mimic significantly increased the level of miR-519d in A549 cells (Figure 4C), and suppressed the expression of HER3 (Figure 4D). In contrast, transfection with miR-519d inhibitor suppressed the miR-519d levels (Figure 4E), and increased the HER3 expression in A549 cells (Figure 4F). These data demonstrate that HER3 is a target gene of miR-519d.

**Figure 4:** **HER3 is a target gene of miR-519d.** (**A**) Identification of conserved miR-519d binding site in 3’-UTR of HER3, using TargetScan. (**B**) Dual luciferase reporter assay showed that miR-519d significantly suppressed the relative luciferase activity of pmirGLO-HER3-3’UTR in 293 cells. (**C**) Real time PCR analysis of miR-519d levels in A549 cells transfected with miR-519d mimic. (**D**) HER3 expression in A549 cells transfected with miR-519d mimics. (**E**) Real time PCR of miR-519d levels in A549 cells transfected with miR-519d inhibitor. (**F**) HER3 expression in A549 cells transfected with miR-519d inhibitor. ^*^p<0.05 vs. control, ^***^p<0.001 vs. control.

### MiR-519d inhibits migration, invasion, proliferation, and survival of A549 cells

To examine the cellular function of miR-519d, we transfected A549 cells with miR-519d mimic or inhibitor, and analyzed the effect on cell migration, invasion, proliferation, and apoptosis. As shown in Figure 5, transfection of miR-519d mimic decreased the HER3 expression and inhibited cell migration and invasion (Figure 5A), while transfection with miR-519d inhibitor increased the HER3 expression and enhanced cell migration and invasion (Figure 5B). In addition, overexpression of miR-519d significantly enhanced A549 cell apoptosis, while inhibition of miR-519d decreased cell apoptosis (Figure 5C).

**Figure 5:** **MiR-519d inhibits A549 cell migration and invasion and induces cell apoptosis.** (**A**) Transfection of miR-519d mimic suppressed the expression of HER3 and inhibited A549 cell migration and invasion. (**B**) Transfection of miR-519d inhibitor increased the expression of HER3 and enhanced A549 cell migration and invasion. (**C**) Upregulation of miR-519d significantly enhanced A549 cell apoptosis, but suppression of miR-519d significantly reduced A549 cell apoptosis. ^**^p<0.01 vs. control, ^***^p<0.001 vs. control.

CCK-8 proliferation assay showed that miR-519d mimic significantly suppressed A549 cell proliferation at 2, 3, 4 and 5 days (Figure 6A), while inhibition of miR-519d increased cell proliferation (Figure 6B). Wound healing assay demonstrated that transfection of miR-519d mimic decreased A549 cell migration capacity, while transfection with miR-519d inhibitor increased A549 cell migration capacity (Figures 6C, 6D). Together, these data show that miR-519d inhibits migration, proliferation, and invasion, and induces apoptosis in lung cancer cells.

**Figure 6:** **MiR-519d reduces A549 cell migration and proliferation.** CCK-8 proliferation assay in A549 cells transfected with miR-519d mimic (**A**), or inhibitor (**B**). Wound healing assay in A549 cells transfected with miR-519d mimic (**C**), or inhibitor (**D**). *p<0.05, **p<0.01, ***p<0.001 vs. as indicated.

### MiR-519d suppresses PI3K/AKT pathway via targeting HER3

HER3 is an important activator of the PI3K/AKT pathway, thereby promoting tumor progression [19]. Hence, we evaluated the effects of miR-519d on the expression of PI3K, p-PI3K, AKT, and p-AKT. Western blot analysis demonstrated that the overexpression of miR-519d significantly inhibited phosphorylation of PI3K and AKT (Figure 7A and 7B). Moreover, suppression of HER3 by siRNA reduced the levels of p-PI3K and p-AKT (Figure 7A). In contrast, suppression of miR-519d enhanced the phosphorylation of PI3K and AKT (Figure 7C and 7D). However, such effects could largely be reversed by silencing HER3 (Figure 7C and 7D). These data indicate that miR-519d suppresses activation of the PI3K/AKT pathway via targeting HER3.

**Figure 7:** **MiR-519d suppresses PI3K/AKT pathway via targeting HER3.** Western blot analyses (**A**) and statistical analysis (**B**) demonstrated that the overexpression of miR-519d significantly inhibited the phosphorylation of PI3K and AKT. (**C**) Suppression of miR-519d enhanced the phosphorylation of PI3K and AKT, but these effects could largely be reversed by silencing HER3. (**D**) Statistical analysis. ^*^p<0.05 vs. control, ^**^p<0.01 vs. control, ^***^p<0.001 vs. control.

### MiR-519d negatively correlates with HER3 in NSCLC tissues

Finally, we examined the HER3 mRNA levels in NSCLC tissues. As shown in Figure 8A, the gene expression of HER3 was upregulated in NSCLC tissues compared to adjacent non-cancerous tissues. Evaluation of the correlation between HER3 and miR-519d gene expression revealed that the miR-519d levels negatively correlate with the HER3 mRNA levels in NSCLC tissues (r=-0.291, P < 0.05) (Figure 8B).

**Figure 8:** **MiR-519d negatively correlates with HER3 in NSCLC tissues.** (**A**) Real time PCR analysis of HER3 mRNA in NSCLC tissues and adjacent non-cancerous tissues. (**B**) Correlation assay showed that miR-519d and HER3 gene expression negatively correlate in NSCLC tissues. **p<0.01 vs. as indicated.

## DISCUSSION

MiRNAs are a group of recently discovered noncoding small RNAs that are approximately 22 nucleotides in length. MiRNAs play an important role in regulating differentiation, proliferation, apoptosis, and metabolism by inhibiting target genes in cells. MiR-519d has been shown to suppress progression of breast cancer and cervical cancer [20, 21]. However, few studies have explored the expression and function of miR-519d in NSCLC patients.

This study demonstrates that both serum and tissue miR-519d levels are significantly decreased in NSCLC patients. The low expression of miR-519d in NSCLC patients was associated with lymph node metastasis and clinical stage, suggesting that the low expression of miR-519d in NSCLC patients may contribute to the invasive nature of non-small cell lung cancer. ROC analysis demonstrated that serum miR-519d levels could be used as a potential biomarker to screen NSCLC patients from healthy controls. Importantly, NSCLC patients with low miR-519d expression had significantly shorter overall survival rates than patients with high serum miR-519d expression. These findings indicate that miR-519d plays a key role in the progression of NSCLC.

We found a conserved binding site for miR-519d in the 3’ UTR of HER3, which is a key regulator in the development of NSCLC. Activation of HER3 was shown to decrease apoptosis, and increase growth and invasiveness of A549 cells [22]. Since our data show that miR-519d inhibition increases HER3 expression and cell migration, these results indicate that HER3 overexpression mediated by miR-519d inhibition plays a key role in promoting migration and invasion of lung cancer cells. However, other target genes related to NSCLC progression might be regulated by miR-519d as well, since miRNAs can have multiple target genes [23]. It will be important to determine in future how many miR-519d-regulated cellular functions are mediated through the repression of HER3, and which miR-519d-regulated functions are not mediated through HER3.

The relationship between HER3, tumor immune tolerance, and the feedback regulation of HER3 in PI3K/AKT signaling pathway are important topics in HER3 research [24]. HER3 regulates the HER2- mediated tumorigenesis, and the expression of HER3 is upregulated in HER2-targeted therapy [24–26]. The increased HER3 expression promotes tumor immune tolerance, which can inhibit the PI3K signaling pathway [27]. HER3 plays a pivotal role between RTK activation and the PI3K/AKT pathway, acts as a negative feedback regulator, and bypasses the activation pathway that leads to immune tolerance against EGFR, HER2 and other targeted therapies [28]. Hence, HER3 has become an important target for tumor therapy.

One of the problems in targeting HER3 in cancer is the lack of effective biomarkers to assess the HER3 activation in patients; this problem also hampers the patients screening [19, 26]. Previous studies have suggested the use of HER3 chaperone kinases (such as HER2) as biomarkers, analysis of HER3 tumor levels using immunohistochemical assays, or using the expression of ligands that activate HER3 as biomarkers [29, 30]. This study is the first to demonstrate that HER3 is a target gene of miR-519d. Our data indicate that miR-519d inhibits activation of the PI3K/Akt signaling pathway via targeting HER3. These results suggest that the HER3 expression in lung cancer tissues is regulated by miR-519d, which may be involved in the development of NSCLC.

However, the present study also has several shortcomings that include the relatively small sample size. In addition, the correlation between HER3 and miR-519d expression needs to be verified in NSCLC tissues. Furthermore, the cellular source of the circulating miR-591d needs to be identified; it will be important to determine whether miR-591d is released only from lung tissues, or from other tissues as well. Future studies should analyze the miR-591d expression in various tissues of NSCLC patients to determine which tissues have the highest expression of miR-591d. Additionally, it will be important to investigate the target tissues of the circulating miR-591d, since this may improve the therapeutic of NSCLC.

In conclusion, our study demonstrates that the miR-519d levels are decreased in serum and tumor tissues of NSCLC patients, and the low miR-519d expression correlates with poor NSCLC prognosis. These data identify the serum miR-519d levels as a potential novel biomarker for NSCLC, and indicate miR-519d regulates the NSCLC progression via targeting HER3.

## MATERIALS AND METHODS

### Patients and specimens

One hundred thirty serum samples from NSCLC patients were collected from the Beijing Luhe Hospital (Beijing, China). The diagnosis of all samples was confirmed by histopathological examination by two pathologists. None of the patients had received neoadjuvant chemo- or radiotherapy before surgery. Based on the classification of malignant tumors by the World Health Organization, the corresponding clinicopathological findings were validated. To define overall survival (OS), the time interval was recorded between the date of surgery and the date of death. Another 50 healthy volunteers, including 24 males and 26 females with an average age of 58.6±14.5 years were enrolled as the normal control group. In addition, a total of 50 lung cancer tissues and 45 adjacent non-cancerous tissues were collected from NSCLC patients who underwent surgery in Beijing Luhe Hospital (Beijing, China) between January 2015 and December 2017. Informed consent was obtained from all participants, and the study was approved by the Ethics Committee of Beijing Luhe Hospital.

### Cell culture

Human A549 and 293 NSCLC cell lines were purchased from the American Type Culture Collection (Manassas, VA, USA). RPMI-1640 medium or DMEM containing 10% fetal bovine serum (FBS) (HyClone, Beijing, China) were used for cell culture at 37°C and 5% CO_2_.

### Transfection

Before transfection, A549 cells were plated at a density of 10^6^cells/well in 6-well plates in 2 ml of DMEM for 24 h. After that, A549 cells were transfected with miR-519d mimics (Guangzhou RiboBio Co., Ltd, Guangzhou, China), and/or HER3 siRNA (Guangzhou RiboBio Co., Ltd, Guangzhou, China) using lipofectamine 2000 (Invitrogen; Thermo Fisher Scientific, Inc.) in accordance with the manufacturer’s protocol.

### Flow cytometry

Annexin V-fluorescein-5-isothiocyanate apoptosis detection kit (BD Biosciences, San Jose, CA, USA) was used to detect the effect of miR-519d on A549 cell apoptosis using BD FACSCalibur system (SKU#: 8044-30-1001, BD Biosciences, Franklin Lakes, NJ, USA). For data analysis, the ModFit software version 4.1 (Verity Software House, Inc., Topsham, ME, USA) was used.

### Luciferase reporter assay

The 3’ untranslated region (UTR) segments containing miR-519d binding sites of HER3 were obtained by PCR. The mutant was cloned using the Fast Mutagenesis System (TransGen Biotech, Beijing, China) according to the instructions. Then, the amplified PCR products were inserted into the pmirGLO Dual-Luciferase miRNA Target Expression Vector (Promega Corporation, Madison, WI, USA). After 293 cells were cotransfected with miR-519d mimic or negative control with recombinant pmirGLO using Lipofectamine 2000 (Invitrogen; Thermo Fisher Scientific, Inc.) for 48 h, Dual-Luciferase Reporter Assay System (Promega Corporation) was used to determine relative luciferase activity according to the instructions.

### RT-qPCR

Total RNA was extracted from serum and tissues of NSCLC patients using the TRIzol reagent kit (Thermo Fisher Scientific, Inc.). For reverse transcription, a TaqMan MicroRNA Reverse Transcription Kit (Applied Biosystems; Thermo Fisher Scientific, Inc.) was used. For qPCR analysis of the relative miR-519d level, SYBR Green Supermix (TaKaRa, Japan) was used according to the instructions. U6 was used as an endogenous control, and the relative gene expression was quantified by the 2^-ΔΔCq^ method [31]. The primers were the following: miR-519d-RT, 5′-GTCGTATCCAGTGCAGGGTCCGAGGTATTCGCACTGGATACGACAAACAGA-3′; U6-RT, 5′-GTCGTATCCAGTGCAGGGTCCGAGGTATTCGCACTGGATACGACAAAATG-3′; miR-519d, forward 5′-CTCCUCCAAAGGGAAGCGC-3'; U6, forward 5′-GCGCGTCGTGAAGCGTTC-3′; universal reverse primer, 5'-GTGCAGGGTCCGAGGT-3'.

### Western blotting

Total proteins were extracted using a total protein extraction kit (Beijing Solarbio Science and Technology Co., Ltd.), and protein concentration was determined by the BCA protein assay kit (Pierce; Thermo Fisher Scientific, Inc.). Western blotting was performed as previously described [32]. The antibodies used were as follows: phosphatidylinositol-4,5-bisphosphate 3-kinase (PI3K; cat. no. 4249, Cell Signaling Technology, Inc., Danvers, MA, USA), phosphorylated (p)-PI3K (cat. no. 13857, Cell Signaling Technology, Inc., Danvers, MA, USA), protein kinase B (AKT; cat. no. 4685, Cell Signaling Technology, Inc., Danvers, MA, USA), p-AKT (cat. no. 4060, Cell Signaling Technology, Inc., Danvers, MA, USA) and GAPDH (cat. no. 5174, Cell Signaling Technology, Inc., Danvers, MA, USA). GAPDH was used as an internal control.

### Immunofluorescence

A549 cells were fixed in 4% paraformaldehyde for 30 min at room temperature (RT). The samples were washed with PBS and incubated with primary antibody against HER3 (1:50 diluted in PBS) in a humidified chamber overnight at 4°C. After that, the slides were incubated with TRITC-conjugated anti-rabbit IgG (1:500 diluted in PBS) mixed with DAPI (1:1000 diluted in PBS) for 20 min at RT. The slides were washed with PBS, sealed, and examined using a fluorescence microscope.

### Cell migration, invasion, and proliferation assays

Cell migration and invasion assays were performed as previous described [33]. Cell proliferation was analyzed using the Cell Counting Kit-8 (CCK8; Dojindo Molecular Technologies, Kumamoto, Japan). Wound healing assay was performed as previously described [33].

### Statistical analysis

The data are presented as the mean ± standard deviation. For comparison of two groups, student’s t-test was used. For comparison of multiple groups, one-way analysis of variance with Fisher's least significant difference test was applied. The Kaplan-Meier method and log-rank test were used to analyze overall survival (OS). To assess whether miR-519d could be used as a potential biomarker, receiver operating characteristic (ROC) curves were used and the area under the curve (AUC) was reported (version 20.0, SPSS, Inc., Chicago, Illinois). P<0.05 was considered statistically different.
